This article has been retracted.

# Application Analysis Based on Big Data Technology in Stroke Rehabilitation Nursing

**DOI:** 10.1155/2021/3081549

**Published:** 2021-12-01

**Authors:** WeiHua Xu, LiangJin Liu, JiuXia Zhang

**Affiliations:** ^1^Department of Neurology, Hubei No. 3 People's Hospital of Jianghan University, Wuhan 430033, China; ^2^Department of Radiology, Hubei No. 3 People's Hospital of Jianghan University, Wuhan 430033, China

## Abstract

According to the statistical analysis, the incidence of stroke disease has gradually increased, particularly in recent years, which poses a huge threat to the safety of human life. Due to the advancement in science and technology specifically big data and sensors, a new research dome known as data mining technology has been introduced, which has the potential value from the perspective of large amount of data analysis. Information has become a new trend of science and technology, and data mining has been used in various application areas to analyze and predict strokes at home and abroad. In this study, big data technology is utilized to collect potential information and explores clinical pathways of level-3 rehabilitation in certain regions of China. Moreover, application effects of data mining in the rehabilitation of patients with the first ischemic stroke have been evaluated and reported. For this purpose, fifty (50) first-time ischemic stroke patients have been screened through big data and were nonartificially assigned to level-3 clinical pathway and conventional rehabilitation groups, respectively, specifically through software. The first group of patients enters the clinical path of the corresponding level according to the way of three-level referral. These patients were analyzed based on the collected results of completing the unified rehabilitation treatment plan of the three-level rehabilitation medical institution in the patient record form. The second group was selected according to the routine rehabilitation model and method of the medical institution where the patients visited were divided into four stages: before treatment, three weeks after treatment, nine weeks after treatment, and seventeen weeks after treatment. For this purpose, a simplified Fugl-Meyer analysis (FMA), recording of various functions of limb movement, and modified Barthel index (MBI) scale were used to analyze and evaluate the ability of daily activities and compare their effects. The final results showed that FMA and MBI scores of the two groups were improved in the three stages after treatment. The FMA and MBI scores of the clinical pathway group on 3rd and 9th weekends were significantly different from those of the conventional rehabilitation group (which is *p* < 0.05). Moreover, difference in FMA and MBI scores between the two at the 17th weekend was not significant. The total cost of the clinical pathway group, particularly at the ninth weekend, was higher than that of the conventional rehabilitation group, but the cost-benefit ratio was better and the incidence of complications was lower than that of the other group.

## 1. Introduction

Every year, approximately 17 million people throughout the world suffer from stroke where 5 million of those patients die and 5 million people have permanent dysfunction or disability, which places a serious burden on the society in general and affected families in particular [1]. At least in the UK, 1.2 million people have had a stroke where 300,000 have moderate to severe disability. About 26% of strokes in the United States have occurred in people under 65 years of age, and an estimated 13 out of 100,000 children have suffered stroke [2]. The burden of stroke is huge for society and individuals. In the UK, the economic loss of stroke is estimated to be 8 billion pounds each year, of which the direct treatment cost of the National Health Service is 3 billion pounds. The cost of informal treatment is 2.4 billion pounds, and the loss of production efficiency is 1.8 billion pounds [3]. The cost of stroke treatment in China is 10 billion yuan each year, which has caused a heavy economic burden on the country. The rate of rehospitalization of stroke patients is significantly higher than that of nonstroke patients [4]. A research report shows that only 15% of stroke patients who survived within 5 years did not undergo rehospitalization [5]. In order to curb the unreasonable growth of medical expenses and improve the utilization of health resources, standardizing the treatment process of diseases is desperately needed. In 1985, the New England Medical Center in the United States took the lead in proposing the concept of clinical pathways. Subsequently, the British National Health Service (NHS) proposed the concept of “clinical management,” developed clinical pathways, and created a clinical pathway user group, called “integrated healthcare pathway.” In September 1996, Singapore Changi General Hospital tried out the clinical pathway project and sent specialists to different hospitals in the United States to conduct training on clinical pathway theory, practice, and management. This was the first clinical pathway in Asia. This working group consisting of doctors, nurses, managers, and related medical staff will plan, implement, and evaluate the transplant clinical pathway management project to the local area. Later, Germany, Japan, and other developed countries successively formulate and manage the clinical pathway. After more than 30 years of practice and development, a relatively complete clinical pathway implementation and management system has been formed abroad. As far as the clinical pathway of stroke is concerned, foreign research is relatively diverse, according to the course of the disease and place of medical treatment. Moreover, the basic principles, program design, service integration, and other perspectives were studied and discussed in clinical pathways [6, 7]. According to the disease course, it is divided into three types: the acute phase of stroke, the rehabilitation phase, and the acute phase and the rehabilitation phase. According to this, the place of medical treatment can be divided into emergency ward stroke clinical pathway, stroke unit clinical pathway, rehabilitation ward clinical pathway, community hospital stroke clinical pathway, and other categories to carry out research [8]. Relatively developed specifically in terms of maturity of the country, the development of clinical pathways in our country has just started and is still in the trial stage.

In this article, we have aimed at “hierarchical and staged rehabilitation medical service institutions,” namely, the rehabilitation medicine department of tertiary hospitals, rehabilitation hospitals, and rehabilitation hospitals. Some of the major contributions of this article are shown in Figure 1.

- The three-level stroke rehabilitation clinical path of community rehabilitation is connected with the clinical path of the acute phase of stroke.
- To shorten the average hospital stay of patients, limit the growth of medical expenses, standardize diagnosis and treatment methods, and strengthen the exchange and cooperation of rehabilitation team personnel.
- Improve the satisfaction of patients and their families and promote the rational use of medical resources. To realize this, we have focused on three levels of stroke rehabilitation in the rehabilitation medicine department of tertiary hospitals, secondary specialist rehabilitation hospitals, and community rehabilitation.
- Finally, significant effects of the clinical pathway on the limb motor function and activities of daily living in patients with stroke in related hospitals in southern Jiangsu and the effect of its application are evaluated.

## 2. Literature Review

Stroke has the characteristics of high morbidity, high mortality, and high disability rate. It is the leading cause of Chinese adult disability. China is a country with a high incidence of stroke. According to the statistics of the Ministry of Health, approximately 2 million new strokes are triggered in China every year. Among these patients, about three-quarters of have varying degrees of dysfunction or disability [2, 3, 9]. The cost of treatment for stroke in China is 10 billion yuan each year, which has caused a heavy economic burden on the country. The rate of later rehospitalization was significantly higher than that of nonstroke patients [4]. A study report showed that only 15% of stroke patients who survived within 5 years did not rehospitalize [5]. One year after the onset, 15–40% of stroke patients lose their upper limb function, 40% have swallowing problems, and 31% have depression. Therefore, many stroke patients need nonprofessional nursing staff (usually family members) to help them complete their daily activities (including bathing, dressing, and getting on the clothes) [10]. This nursing burden seriously affects the physical and mental health of nursing staff. According to statistics, up to 48% of nursing staff have health problems, and two-thirds have a significant decline in quality of life [11].

In 1980s, the New England Medical Center in the United States took the lead in proposing the concept of clinical pathways to standardize the disease treatment process, improve the utilization of health resources, and curb the growth rate of medical expenses. Subsequently, the British National Health Service (NHS) proposed “clinical management” (clinical governance) concept to develop clinical pathways and create a clinical pathway user group, called “integrated care pathway” (ICP). In September 1996, Singapore Changi General Hospital tried out the clinical pathway project and sent specialists to different hospitals in the United States to conduct training on clinical pathway theory, practice, and management. This is the first attempt in Asia to try the clinical pathway. This is a work group composed of doctors, nurses, managers, and related medical personnel for transplantation. Clinical pathway management projects were planned, implemented, and evaluated locally. Afterwards, developed countries such as Germany and Japan successively carried out a lot of research and exploration on the formulation and management of clinical pathways. After more than 20 years of practice and development, foreign countries have formed a relatively complete clinical pathway implementation and management system. As far as the clinical pathway of stroke is concerned, foreign studies are relatively diverse and relatively mature. The clinical pathways are studied from various perspectives such as the course of the disease, the place of medical treatment, basic principles, program design, and service integration. Discuss [6, 7], where the course of disease is divided into three categories: acute stroke clinical path, rehabilitation phase clinical path, acute phase, and rehabilitation phase clinical path [8]; the place of medical treatment is based on the clinical path of stroke in the emergency ward; stroke unit clinical pathways, rehabilitation ward clinical pathways, and community hospital stroke clinical pathways have been studied in various categories, but there is no unified conclusion. Some studies believe that clinical pathways can significantly reduce the length of stay and cost of stroke patients [12, 13]. Additionally, various studies believe that clinical pathways increase the number of days of hospitalization of patients [14, 15].

The research on clinical pathways in China, its research methods, research angles, and evaluation indicators are similar to those of foreign countries, and most of these are based on advanced foreign experience. Foreign research objects are mainly based on multiple medical institutions to explore the role of clinical pathways. Most domestic research studies on the clinical pathways of stroke from the perspective of nursing mainly study the effect analysis of clinical nursing pathways in a certain hospital. This is also different from the domestic and foreign medical systems, severity of the disease, and differences in treatment. Moreover, it is more feasible to explore the application of clinical pathways of stroke from the perspective of nursing. Most domestic reports on the effects of clinical pathways of stroke are mainly positive reports, and there are few negative reports. If more, it can effectively promote the patient's limbs, rehabilitation, reduction of hospitalization days, reduction of hospitalization costs, and improvement of patient satisfaction, etc. It may be currently in a critical period of medical system reform, and it is necessary to report positively promoting the application of clinical pathways. Although a clinical pathway treatment system for stroke has also been established in China. However, most of them are mainly based on the clinical pathways in the acute phase of stroke and the clinical pathways in the recovery phase of stroke, aiming at the treatment design in stroke units and rehabilitation wards, and lack of relevant clinical pathways in community hospitals, and lack of continuous hierarchical levels, and clinical path of stroke rehabilitation at different stages.

The personal response and recovery of nerve injury after stroke are complex and changeable. This requires not only the cooperation of emergency physicians, neurologists, and nurses but also the cooperation of personnel from multiple disciplines, such as rehabilitation physicians and physical therapists, teachers (PT), occupational therapists (OT), speech and language therapists (SALT), and nursing workers, by providing their knowledge and professional skills to benefit stroke patients. A review of the literature, as well as the analysis of quantitative and qualitative research data related to improving the recovery after stroke, demonstrated that different levels of medical staff have different intervention times for the clinical path of stroke, different treatment modes, and different contributions to improving rehabilitation after stroke. It is mainly reflected in three stages, namely the first stage, the acute stage of rehabilitation; the second stage, the inpatient rehabilitation; and the third stage, the rehabilitation after discharge.

The first phase, acute rehabilitation. In the National Stroke Strategy for England, Wales, and Northern Ireland, 6 out of 22 quality standards clearly emphasize the early intervention of rehabilitation professionals, providing professional skills and knowledge to improve the quality of treatment and improve patient outcomes. There is clear evidence that shows that a multidisciplinary team with the cooperation of rehabilitation therapists is significantly more effective for stroke hospitalization. This study evaluates all previous randomized trials and has rehabilitation treatment. A comparison of the comprehensive stroke unit cooperated by the teacher with the treatment effect in the traditional medical ward (21 trials, 3994 participants) proves that the former reduces the mortality rate and the patients receiving comprehensive rehabilitation treatment are more independent; this advantage is in stroke that persists within one year of living at home after being discharged from the hospital. Therefore, regardless of age, gender, disability, and the severity or type of stroke, multidisciplinary treatment involving rehabilitation professionals in stroke treatment is to provide high-quality brain stroke treatment.

The second phase, inpatient rehabilitation. Stroke inpatient rehabilitation usually refers to professional stroke rehabilitation institutions, including rehabilitation doctors, rehabilitation nurses, physical therapists, occupational therapists, speech and language therapists, and assistants. In most National Health Service agencies, dietitians, clinical psychologists, and social workers are not unit-based and work more on the periphery. Patients are usually evaluated early within 24 hours and are based on national clinical guidelines, and the Sentinel National Stroke Plan standard provides appropriate referrals to ensure that these professionals assist in recovery when specific needs are identified.

In most countries, inpatient stroke rehabilitation is supported by evidence-based national clinical guidelines and relies on rehabilitation teams to plan, provide, and evaluate treatment. Langhorne [16] believes that the treatment that is most likely to improve the final outcome intervention is repetitive rehabilitation training, focusing on clarifying the needs of stroke patients and inducing them to complete related exercise therapy. Physiotherapy, occupational therapy, and speech and language therapy interventions can improve the outcome of stroke patients, but the mechanism of action and the most effective intervention of the format have not yet been determined. Legg et al. [17] found in 9 randomized controlled studies (1,258 participants) that OT treatment increased the ability of daily living (ADL) score and reduced the probability of poor prognosis . In order to improve ADL patients, one in eleven patients has a good prognosis. Brady [18] completed a retrospective study of patients with aphasia after stroke, mainly for these patients who received speech and speech therapy. The entire study included 39 randomized controlled studies (2,518 participants). The study determined some evidence that proved the effectiveness of SALT in improving communication skills and accepting language skills in patients with aphasia after stroke. However, Brady et al. concluded that the current evidence is insufficient to conclude that one specific SALT intervention is more effective than another. Similarly, in more discussions on post-stroke rehabilitation methods, Pollock [19] include 96 studies (10,401 participants) concluded that rehabilitation therapy, including partial rehabilitation therapy, is effective in restoring functions and activities after stroke. In view of the results of these studies, we need to establish a unified clinical pathway and adopt a method consistent with evidence-based basis for rehabilitation training, so that all stroke treatment teams can improve the ADL of stroke patients and enhance their function and mobility and communication skills.

The third phase is rehabilitation after discharge (community rehabilitation). It must be realized that the treatment of stroke cannot be indefinite by specialist doctors. Although stroke patients and their caregivers have clear long-term medical support demand, there is currently little information on how to better support treatment. The expert consensus is that once the rehabilitation goal is reached, the treatment plan may be taken over by a nonprofessional, community-based medical institution. This reflects a point of view that stroke treatment varies according to the needs of patients, and in stroke community rehabilitation, what medical staff need most is knowledge and understanding of community rehabilitation treatment, not stroke specialist knowledge. Currently proposed by the UK, all stroke patients should be followed up regularly within 6 months after the illness. Although the background and implementation of this plan are not specified, and the current implementation is not complete, stroke patients need some form of longer-term follow-up. The treatment has been recognized. Self-management is increasingly seen as the most appropriate way for patients who need long-term support, and it has now become part of helping people adapt to life after stroke. This adjustment takes time and, therefore, requires to develop a staged clinical path of stroke through the education and support of stroke patients and their families. In later stage of inpatient rehabilitation treatment, patients will be less dependent on professional rehabilitation personnel. They will be more able to understand and manage themselves, so that stroke patients can become self-conscious.

## 3. Proposed Big Data-Enabled Method

Around fifty (50) cases of ischemic stroke patients, specifically those who were hospitalized in the Department of Rehabilitation Medicine of a University Hospital in China from January 2013 to January 2015, were screened through the big data and divided into clinical pathway (25 cases). Furthermore, routine groups were divided according to the random number table method rehabilitation groups (25 cases). The possible selection criteria are based on the following:

1. Meet the diagnostic criteria of the Chinese Guidelines for the Diagnosis and Treatment of Acute Ischemic Stroke, and it was confirmed as the first onset by CT or MRI.
2. Age 45–75 years.
3. Course of disease 7–15 days.
4. Clear consciousness, GCS ≥13 points.
5. Cognitive function.

MMSE (illiterate) ≥18 points; MMSE (primary school) ≥ 21 points; MMSE (middle school including technical secondary school) ≥23 points; MMSE (university) ≥24 points; (6) severity of neurological impairment: National Institutes of Health Stroke Scale (NIHSS) ≤16 points; (7) moderate to severe motor dysfunction: simplified Fugl-Meyer motor function <85 points; (8) if the patient at the same time accompanied by other diseases, no special treatment is required during the hospitalization and does not affect the implementation of the clinical pathway process of the first diagnosis; (9) all patients have signed the informed consent.

Exclusion criteria:

1. A history of cerebral infarction of two or more times.
2. Severe clinical complications or complications: severe liver and kidney disease, decompensated heart insufficiency, heart or respiratory arrest or myocardial infarction within 3 months, severe pneumonia or chronic obstructive pulmonary disease, deep vein thrombosis, etc.
3. Other diseases or medical history that affect motor function, such as a history of fractures of limb dysfunction on the side of hemiplegia, amputation, and history of lower limb osteoarthritis that affects walking, malignant tumors, pregnancy, etc.
4. Suffering from severe mental illness or accompanied by mental symptoms.
5. Severe aphasia, which affects communication and cannot cooperate with examinations and rehabilitation training.
6. Those who have not signed an informed consent based on big data records. There is no difference in gender, age, course of disease, and hemiplegia between the two groups. *p* > 0.05 is considered statistically significant as depicted in Table 1.

### 3.1. Proposed Methods

#### 3.1.1. Clinical Pathway Group Method

According to the patient files recorded by the big data, select the patients in the clinical path group and then perform comprehensive index evaluation according to the unified rehabilitation treatment plan of the three-level rehabilitation medical institution in the record, that is, the rehabilitation medicine department of the tertiary general hospital (the number of hospitalization days is 3 weeks), second-level specialist rehabilitation hospitals (6 weeks of stay in hospital), and community rehabilitation institutions (family rehabilitation guidance for 8 weeks). According to big data, it takes 17 weeks for the clinical pathway group to complete a set of three-level referrals. The clinical pathway group rehabilitation training requirements are given as follows:

1. Department of Rehabilitation Medicine in a tertiary general hospital: the standard hospital stay is 20-21 days (3 weeks). After acute clinical treatment (usually about 1–2 weeks), select the corresponding one based on the patient's rehabilitation evaluation results. Class-level rehabilitation program. Specific items include exercise therapy training; occupational therapy, corresponding speech and swallowing therapy for patients with speech and swallowing disorders, physical factor therapy, and traditional Chinese medicine rehabilitation therapy. Specific time requirements: exercise therapy training and homework. The daily training time totals 1.5 hours, of which the exercise therapy training intensity is 60 minutes a day, and other additional training time can be appropriately increased depending on the patient's tolerance; the daily training time of swallowing function is 70 minutes in total, of which the manual training intensity is 30 minutes a day, neuromuscular electrical stimulation is 2 times a day, 20 minutes each time, and other additional training time depends on the patient's tolerance and can be increased appropriately; speech function training time: training intensity 30 minutes a day, other additional training time depends on the patient's tolerance level that can be increased appropriately; nursing education and psychological counseling: according to the content of nursing records, 1 time/day; depending on the needs of the patient, increase appropriately during admission and discharge.
2. Second-level specialist rehabilitation hospitals: standard hospitalization days are 40–42 days ((6 weeks). According to the patient's rehabilitation assessment results, select the corresponding second-level rehabilitation program. The specific items are the same as those of the rehabilitation medicine department of a third-level general hospital. Specific time requirements: exercise therapy training and occupational therapy, a total of 3 training hours per day; the exercise therapy training intensity is 90 minutes a day, and other additional training time can be appropriately increased depending on the patient's tolerance; the training schedule of swallowing function and speech function is the same as that of the rehabilitation department of tertiary general hospitals; nursing education and psychological counseling: according to the contents of the nursing records, 1 time/day, depending on the needs of the patient during admission and discharge.
3. Community rehabilitation organization (family rehabilitation guidance for 8 weeks). Patient rehabilitation records were collected based on big data, which follow the family training program record form. It is required to formulate a corresponding weekly training program, and it is required to complete the content of the family training program once a day, and the training time is not less than 60 minutes a day. During the implementation process, the opinions of patients and their families are solicited, with a view to continuous modification and supplementation.

#### 3.1.2. Conventional Rehabilitation Group Method

The treatment content records of the conventional rehabilitation group were collected by big data while ensuring that the basic conditions at the time of enrollment are consistent with the clinical pathway group. Moreover, the experimental process is completed according to the conventional rehabilitation mode and method in the current three-level rehabilitation institutions and standard hospitalization days and rehabilitation treatment. There are no restrictions on the content and treatment time and intensity, but the treatment content and time need to be truthfully recorded in the rehabilitation treatment record sheet, recorded once a week for a total of 17 weeks of follow-up.

### 3.2. Evaluation Method

Experimental results are completed by the same evaluator, who has been trained in the training process. Evaluators will not participate in the enrolled patients' rehabilitation treatment and other test processes except for the evaluation. They will be conducted at the beginning of the treatment, on the 3rd weekend after the treatment, the 9th weekend, and the 17th weekend. Evaluation. The simplified Fugl-Meyer motor function scale is used to evaluate motor function of the limbs, which is divided into total scores, i.e., upper limb and lower limb scores, respectively. For muscle reflex, flexor and extensor coordinated movement, activities accompanied by coordinated movement, activities that depart from coordinated movement, and reflexes. The hyperactivity, joint stability, coordination ability, and speed are scored. Each item is worth 0∼2 points, and the total score is calculated; The hyperactivity, joint stability, coordination ability, and speed are scored. Each item is worth 0∼2 points, and the total score is calculated; the modified Barthel index scale is used to assess the patient's activities of daily living, according to toileting, eating, urinating and defecation control, bed and chair transfer, level walking, and other 10 content items, each item is given 0–15 points, and the total score is calculated. On the 9th weekend after treatment, compare the total hospitalization and rehabilitation costs of the two groups as well as the required costs and MBI and increase the ratio of points.

### 3.3. Complication Indicators

According to the patient records collected by big data, at the 9th week after treatment, the two groups of complications were compared, including pulmonary infection, urinary tract infection, lower extremity venous thrombosis, shoulder-hand syndrome, and pressure ulcers. Lung infection by auscultation and chest lung lobe imaging changes on film examination are the criteria. Urinary tract infections are determined by urinary tract irritation and positive mid-level urine culture as the criteria. Lower limb venous thrombosis is the presence of lower limb swelling and pain. B-ultrasound changes in vascular imaging are the criteria. Shoulder-hand syndrome is based on pain, swelling, and restricted movement in the shoulder and hand on the hemiplegic side, and X-rays and related examinations have excluded other causes. The criterion for pressure skin ulcers is the appearance of skin ulcer at the compressed site.

### 3.4. Statistical Analysis

Statistical software was used to analyze the data, which were expressed as the mean ± standard deviation (*x* ± *s*). The paired-sample *t*-test was used for comparison within groups, and the independent sample *t*-test was used for comparison between groups. The homogeneity of variance was performed before the *t*-test. If variance is uniform, then use the t and rank sum tests for statistical analysis. *p* < 0.05 considers the difference to be statistically significant.

(1) $$\begin{array}{c} \sigma =\sqrt{\frac{1}{N}\sum_{i=1}^{n}{\left(x_{i}-\mu \right)}^{2}},\\ s=\frac{\sigma }{\sqrt{n}}. \end{array}$$

## 4. Experiments and Results

In order to verify various claims of the proposed big data-based model, different experiments were carried out in the real environment of hospital where the number of patients and treatment plans were based on the proposed model. In this section, a detailed comparative analysis of the proposed and existing state of the art methods is presented.

### 4.1. Function Improvement

According to the treatment of two groups recorded by big data, particularly before treatment, difference in FMA and MBI scores between the clinical pathway group and conventional rehabilitation group was not statistically significant (*p* > 0.05). Compared with the pretreatment within the group, FMA and MBI scores of two groups increased gradually on the 3rd weekend, 9th weekend, and 17th weekend after treatment, and difference was statistically significant (*p* < 0.05). At the 3rd weekend after treatment, MBI score was significantly higher than that of the conventional rehabilitation group (*p* < 0.05). At the 17th weekend after treatment, there was no significant difference in FMA and MBI scores between the clinical pathway group and the conventional rehabilitation group (*p* > 0.05) as shown in Table 2 and Figures 2–4.

### 4.2. Treatment Expenses

During the treatment of two groups of patients, total hospitalization expenses and rehabilitation expenses of the clinical pathway group from the start of enrollment to the 9th weekend after treatment were significantly higher than those of the conventional rehabilitation group, and the comparison was statistically significant (*p* < 0.05). See Table 3 and Figure 5. Comparing the MBI scores of the previous two (the 9th weekend after treatment and before treatment), for every increase of 1 point in the MBI score, the total hospitalization and rehabilitation expenses of the clinical pathway group are lower than those of the conventional rehabilitation group, and the comparison between the two is statistically significant (*p* < 0.05).

### 4.3. Complications

During the treatment of two groups of patients, the clinical pathway group had 3 cases of pulmonary infection, 2 cases of urinary tract infection, 0 cases of lower limb venous thrombosis, 1 case of shoulder-hand syndrome, and 0 cases of pressure sores in the clinical pathway group from the beginning of the group to the 9th weekend after treatment. In the conventional rehabilitation group, there were 5 cases of pulmonary infection, 3 cases of urinary system infection, 1 case of lower limb venous thrombosis, 3 cases of shoulder-hand syndrome, and 1 case of pressure ulcers. All patients improved after symptomatic treatment, and there were no deaths in both groups. The overall complication rate of patients was 24.0% and 52.0%, and the difference between the two was statistically significant (*p* < 0.05), which is shown in Figure 6.

The results show that with the extension of treatment time, the FMA and MBI scores of the two groups increased significantly compared with the previous time point, suggesting that whether it is the clinical pathway group or the conventional rehabilitation group, tertiary rehabilitation treatment can effectively improve the motor function of the limbs and activities of daily living of stroke patients. The FMA and MBI scores of the clinical pathway group were significantly higher than those of the conventional rehabilitation group on the third weekend and the ninth weekend after treatment. It can more effectively improve the motor function and ability of daily living of stroke patients and improve the quality of rehabilitation. However, after the patient enters the community or home to receive rehabilitation treatment at the 17th weekend after treatment, there is no significant difference between the FMA and MBI scores of the two groups. Explain that when it comes to the third-level rehabilitation stage, that is, the community or family rehabilitation stage, because it is only pure rehabilitation education or guidance, the patient does not go to a special rehabilitation institution, does not have professional rehabilitation personnel on-site guidance and supervision, and cannot be completed as required. Their athletic ability and the ability of activities of daily living have not been further improved, which may also indicate that the curative effect of the tertiary rehabilitation clinical pathway lasts for less than 17 weeks.

## 5. Conclusion

In recent years, as China's economic development has continued to accelerate, comprehensive national strength continues to increase and the country's investment in medical resources has gradually increased. China's tertiary rehabilitation network has continued to strengthen, and tertiary first-class hospitals have established rehabilitation medicine departments and second-level specialist rehabilitation hospitals. Community rehabilitation centers and other institutions have gradually increased. From the perspective of the rational deployment of medical resources, stroke patients have a very large demand for community rehabilitation, but it is currently difficult to meet. Patients perceive a doctor between different levels of rehabilitation institutions, and there is no unified referral and rehabilitation treatment system standard that can be used for reference. In order to make the three-level rehabilitation system for stroke patients as effective and cost-effective as possible, it is imperative to establish a unified referral process and rehabilitation plan.

In this study, we have designed a big data technology-based information collection system specifically for stroke patients based on the original three-level rehabilitation, which are treated in a hospital in a certain region of China. It compares changes in FMA and MBI scores of the clinical pathway group and conventional rehabilitation group, as well as the related costs. In order to meet the precision rehabilitation, the requirement is to provide individualized rehabilitation treatment for dysfunction. The ultimate goal is to actively improve the patient's various functions and activities of daily living, and help the patient return to a normal society and family life as soon as possible. On the basis of conventional rehabilitation treatment for patients with ischemic stroke, the implementation of the three-level rehabilitation clinical path can promote the patient's limb motor function and better recovery of the ability of daily living in the early stage, and improve the patient's quality of life. It is worthy of further research and promotion. In the later stage or in community or family rehabilitation training, it is necessary to encourage and guide patients to persist in training according to the requirements of the path and at the same time to do a good job in the training of relevant rehabilitation knowledge for family members, to play its role in supervision and assistance, and to enhance patient confidence, so that patients can take care of themselves and return to life. A normal social life lays the foundation. It is very important for patients who return to their families or communities after inpatient rehabilitation treatment to enter a standardized community rehabilitation system to receive rehabilitation treatment.

## Figures and Tables

**Figure 1:** Area of origin of stroke.

**Figure 2:** FMA scores of the two groups of patients before and after treatment.

**Figure 3:** MBI scores of two groups of patients before and after treatment.

**Figure 4:** MBI *t* and *p* values of two groups of patients.

**Figure 5:** Cost *t* and *p* values of two groups of patients in the 9th week.

**Figure 6:** Comparison of the number of complications between two groups.

**Table 1:** General information of the two groups of patients.

Groups	Numbers	Man	Woman	Ages	Course of disease
Clinical	25	13	12	62.52 ± 7.65	9.52 ± 2.26
Regular	25	15	10	62.20 ± 7.44	9.72 ± 2.89

**Table 2:** FMA *t* and *p* values of two groups of patients.

Item	Before treatment	3 weekends after treatment	9 weekends after treatment	17 weekends after treatment
*t*	0.457	2.028	2.342	1.992
*p*	0.650	0.048	0.023	0.052

**Table 3:** Cost of 9th week of treatment for two groups of patients.

Groups	Total cost	Recovery fee	Total cost/BMI	Recovery fee/BMI
Clinical	57327	20485	1450	521
Regular	44216	15264	2092	757

## Data Availability

The datasets used and analyzed during the current study are available from the corresponding author upon reasonable request.
